The article "Peanut-Related Perforated Diverticulitis Before the Age of 60" was published in 2021. Journal: Cureus.

# Peanut-Related Perforated Diverticulitis Before the Age of 60

**DOI:** 10.7759/cureus.19767

**Published:** 2021-11-20

**Authors:** Charles K Lee, Christopher A Wisnik, Ameen Abdel-Khalek, Orlando Fleites, Stephanie S Pelenyi, Ammarah Tariq, Frederick Tiesenga

**Affiliations:** 1 Medicine, Saint James School of Medicine, Park Ridge, USA; 2 Surgery, West Suburban Medical Center, Oak Park, USA; 3 Medicine, Poznan University of Medical Sciences, Poznan, POL; 4 Anesthesia, Avalon University School of Medicine, Willemstad, CUW; 5 General Surgery, West Suburban Medical Center, Oak Park, USA

**Keywords:** complicated diverticulitis, exploratory laparotomy, sigmoid resection, sigmoid diverticulitis, diverticular disease

## Abstract

We present a case in which a 55-year-old male with a past medical history of systemic lupus erythematosus (SLE) and rheumatoid arthritis (RA) presented with sharp, worsening right-sided abdominal pain radiating across the entire abdomen after eating peanuts. Computed tomography (CT) imaging showed evidence of acute sigmoid diverticulitis complicated by a walled-off perforation. The patient’s past medical history suggested previous recurrent episodes of diverticulitis. Our patient underwent exploratory laparotomy, sigmoid colon resection with low anterior anastomosis and proctocolectomy, and loop ileostomy. During treatment, the sigmoid colon was found to be very indurated and abnormally going all the way down to the peritoneal reflection. Appropriate identification of the patient’s condition and timely intervention resulted in a successful outcome.

## Introduction

Diverticulitis is inflammation of one or more diverticula, which are outpouchings of the colon. Together with diverticulosis (the formation of diverticula), diverticulitis is described under the umbrella categorization of diverticular disease, but is more technically identified as symptomatic diverticulosis [1]; approximately 15%-20% of diverticulosis are symptomatic, i.e. become inflamed and transform into diverticulitis [2]. Risk factors for diverticular disease include advanced age (in the United States, almost 80% of individuals over the age of 85 years are estimated to be affected by diverticular disease [3]), immunodeficiency (for instance due to medical management of autoimmune conditions), and lifestyle factors such as a diet low in fibers and high in red meat [2,4-7].

Obstruction of diverticula and inflammatory processes are thought to be a part of the pathophysiology of diverticulitis [8], and research has also shown that diverticula form at areas of weakness in the gut wall which are susceptible to herniation but are also thinner due to muscle layer atrophy [8,9], which predisposes these areas to perforation not just by inflammatory processes but luminal trauma by a variety of items including foreign bodies and ingested items [10,11]. Traditionally, patients at risk for or diagnosed with diverticular disease were recommended to avoid hard foods such as nuts (including peanuts), seeds, corn, and popcorn [12,13] for concerns of entrapment and perforation by mechanisms such as luminal trauma.

The article "Peanut-Related Perforated Diverticulitis Before the Age of 60" was published in 2021. Journal: Cureus.

Diverticulitis is a clinical diagnosis; work-up typically includes CT imaging, a determination as to whether the diverticulitis is complicated or uncomplicated, and if uncomplicated, a determination of whether or not the patient meets systemic inflammatory response syndrome (SIRS) criteria [5]. Uncomplicated diverticulitis is localized diverticular inflammation, whereas complicated diverticulitis is diverticular inflammation with an abscess, phlegmon, fistula, obstruction, bleeding, or perforation [5,7]. The SIRS criteria requires meeting at least two of the following four conditions: temperature greater than 100.4°F or less than 96.8°F; heart rate greater than 90 beats per minute; respiratory rate greater than 20 breaths per minute or PaCO2 less than 32 mm Hg; white blood cell count of greater than 12,000 per mm2, less than 4,000 per mm2, or more than 10% band forms [5]. Cases of diverticulitis that are complicated are managed by surgery, or percutaneous drainage if the complication is an abscess [5-7], regardless of SIRS criteria. Patients with uncomplicated diverticulitis and who do not meet SIRS criteria are typically not admitted but usually sent home with instructions for a course of antibiotics for 7-10 days and a clear liquid diet for 2-3 days; patients with uncomplicated diverticulitis who meet SIRS criteria are admitted, placed on IV antibiotics, and made nil per os (NPO, meaning no oral intake). Admitted patients with uncomplicated diverticulitis that fail to improve with IV antibiotics are managed by urgent colectomy with end colostomy [5].

Here we discuss the case of a 55-year-old male with a past medical history of systemic lupus erythematosus (SLE), rheumatoid arthritis (RA), and suggestive of recurrent diverticulitis presenting with sharp right-sided abdominal pain radiating across the entire abdomen after eating peanuts; he was found to have evidence of acute sigmoid diverticulitis on CT with evidence of a walled-off microperforation, making his condition a complicated diverticulitis.

## Case presentation

Chief complaint

Our patient is a 55-year-old male reporting sharp right-sided abdominal pain with onset one day prior to presentation.

History of present illness

The patient had seen his primary care physician for constipation 11 days prior to admission, which was treated with polyethylene glycol 3350 (MiraLAX, Braintree Laboratories Inc., Braintree, MA, USA) at the time. The patient reports that his symptoms started suddenly on the day prior to the presentation which was preceded by a large, soft bowel movement. The patient denied any associated chest pain, shortness of breath, fevers/chills, cough, or any other signs of infection. The patient presented to the emergency department because he was unable to get an appointment with his primary care physician. The patient also reported eating peanuts (which he consumes frequently) on the day prior to presentation.

The article "Peanut-Related Perforated Diverticulitis Before the Age of 60" was published in 2021. Journal: Cureus.

Past medical history

The patient’s past medical history includes a deep venous thrombosis (DVT) in his left leg over 20 years ago, coagulopathy controlled by warfarin, SLE, and RA; both autoimmune conditions (SLE and RA) are controlled by hydroxychlorquine. Of note, the patient also reported that he had similar sharp, stabbing pains in the past, most recently at his last appointment with his primary care physician; the most recent of these pains spontaneously resolved with daily MiraLAX intake. The patient has never smoked tobacco.

Examination

On examination, the patient was found to have mild lower abdominal tenderness without rebound, but the examination was otherwise unremarkable.

Investigations

While in the emergency department, the patient underwent a CT scan, which showed acute sigmoid diverticulitis with a walled-off perforation, making the patient’s diverticulitis a complicated diverticulitis (Figure 1). The perforation was suspected to be a microperforation, but as the patient did not appear acutely toxic, consultations were made with other specialists to discuss the possibility of bowel resection after the resolution of the patient’s acute symptoms. During his entire inpatient stay, the patient’s white blood cell count remained low and stable.

**Figure 1:** Abdominal CT (coronal) showing bowel wall thickening and small foci of gas next to the sigmoid colon suggestive of perforation.

Preoperative diagnosis

Based on the patient’s history, associated investigations, and imaging, the preoperative diagnosis was complicated diverticulitis.

Treatment

The patient underwent an exploratory laparotomy, sigmoid colon resection with low anterior anastomosis and proctocolectomy, placement of two Jackson-Pratt (JP) drains, and loop ileostomy. Notable pathology during the operation consisted of a very indurated abnormal sigmoid colon going all the way down to the peritoneal reflection, which was dissected out. The descending colon was transected above the level of inflammation with a gastrointestinal anastomosis (GIA) stapler (US Surgical Corp., Nonvalk, CT, USA) and then the affected colon was dissected out along its mesenteric attachments with Sonicision (Covidien, Mansfield, MA, USA) below the level of the chronic inflammation. After this, it was transected with a thoracic-abdominal (TA) stapling device (US Surgical Corp., Nonvalk, CT, USA) and the removed portion of the colon was sent to pathology for further analysis for possible neoplasia. Due to the very low nature of the anastomosis, it was decided to perform a diverting loop ileostomy.

The article "Peanut-Related Perforated Diverticulitis Before the Age of 60" was published in 2021. Journal: Cureus.

Post-operative diagnosis

The postoperative diagnosis was complicated diverticulitis.

Outcome/progress

After recovering from anesthesia, the patient was followed for four days in an inpatient setting, the course of which was uneventful. Samples sent to pathology from the operation were negative for tumors but revealed multiple diverticula and a serosal abscess cavity measuring 3.2 x 2.6 x 1.1 cm which was filled with green-yellow pus. The patient was discharged home on the fourth postoperative day and followed in an outpatient setting. In the outpatient clinic follow-up eight weeks after his procedure, the patient reported complete resolution of his symptoms.

## Discussion

Diverticular disease is traditionally taught and understood as a condition of the elderly (i.e. over 65 years of age), and known risk factors include advanced age, obesity, immunodeficiency, and diets that are low in fiber and high in fat and/or red meat [2,4-7]. Of these, age is typically considered the most prognostic factor [2,4,14]; acute diverticulitis is uncommon in patients under the age of 40 and typically occurs in patients over the age of 60 [15]. However, recent research has observed an increasing trend of hospital admissions in the United States for diverticulitis and diverticular disease for patients under the age of 60 [16-18]. This trend has not been limited to the United States; at least one study of an Italian population has found a similar trend of more individuals younger than the traditional age range for diverticular disease being admitted for diverticulitis, a majority of these individuals being male [19]. Further, some research has suggested a seasonal or sinusoidal pattern for diverticulitis admissions in the United States, with a peak during the summer months [20]. A number of studies suggest that the traditional understanding of diverticulitis and its management need updating to accommodate more recent research suggesting an increased rate of diverticulitis among individuals under the age of 65, and that diverticulitis management should be based on disease severity rather than the age of the patient [4,7,8,17-19,21].

The article "Peanut-Related Perforated Diverticulitis Before the Age of 60" was published in 2021. Journal: Cureus.

Among the traditional recommendations for patients at risk for or diagnosed with diverticular disease was avoidance of hard foods such as nuts (including peanuts), seeds, corn, and popcorn [12,13]. However, recent research such as the study by Strate et al. (2008) suggests that nut, corn, and popcorn consumption is not associated with an increased risk of diverticular disease or complications thereof [13]. As a result, these and other sources advise against avoiding foods such as nuts and seeds, asserting that there is little or no evidence in the literature to support the traditional recommendation [12,13,22,23]. However, these sources are unable to address certain aspects of the physical mechanics that underlie diverticula formation, notably that diverticula occur at areas of weakness in the gut wall [8,9], predisposing these areas to perforation not just by inflammatory processes but also luminal trauma by a variety of items including both foreign bodies and ingested items [10,11]. Therefore, these sources, as Strate et al. themselves observe, are unable to rule out luminal trauma from hard foods such as nuts as a cause of diverticular perforation [23].

Of the traditional risk factors for diverticular disease, our patient has one (immunodeficiency), but other circumstances of his case are consistent with some recent research related to diverticulitis presentations in that he is younger than the age ranges typically associated with diverticulitis, is male, and was admitted in a summer month (August). In contrast with other recent research, however, the mechanisms by which our patient developed diverticulitis at an age earlier than typical presentations may also be related to his high peanut consumption. Based on the findings in our case, particularly the multiple diverticula present in the sigmoid colon resected from our patient, it is likely that our patient’s sigmoid colon wall was weakened and compromised well before, potentially years before, the onset of episodic pain. It is possible that the onset of symptoms in our patient was precipitated by luminal trauma to an already-compromised colon wall by frequent peanut consumption. The walled-off nature of our patient’s perforation may have contributed to relief of symptoms in the past with daily MiraLAX intake. In addition, the recurrent episodes of flare-ups of pain may have also been due to disturbance of the walled-off perforation by the passage of hard foods such as peanuts.

The management of our patient was based on imaging findings, physical examination, and patient history, and in spite of his younger age and autoimmune conditions, he was managed and treated in an appropriate and timely manner, resulting in a successful outcome.

The article "Peanut-Related Perforated Diverticulitis Before the Age of 60" was published in 2021. Journal: Cureus.

## Conclusions

Diverticulitis, i.e. symptomatic diverticulosis, was traditionally considered a condition of the geriatric population over the age of 65 years but is also associated with other risk factors, including a high-fat/red meat diet and immunodeficiency. However, some recent research has shown a marked increase in hospital admissions for diverticulitis in individuals under the age of 60 years in the United States, many of whom lack the other traditionally associated risk factors as well. Other recent research has failed to support the traditional recommendation that individuals with or at risk of diverticular disease avoid certain hard foods such as nuts (including peanuts), seeds, corn, and popcorn; these sources, however, do not account for the physical mechanisms underlying the pathophysiology of diverticular perforation and are therefore unable to rule out luminal trauma due to passage of hard foods and other substances as a mechanism of diverticular perforation. Our case demonstrates the need to appropriately diagnose and manage diverticulitis in any population, regardless of age, and also demonstrates a possible mechanism by which the traditional recommendations for diverticular disease may remain valid for patients with risk factors for diverticular disease such as autoimmune conditions treated by medications with immunosuppressant effects.
